# Risk Factors and a Nomogram Model Establishment for Postoperative Delirium in Elderly Patients Undergoing Arthroplasty Surgery: A Single-Center Retrospective Study

**DOI:** 10.1155/2021/6607386

**Published:** 2021-12-02

**Authors:** Daiyu Chen, Ying Li, Qingshu Li, Wuxi Gao, Jiaoni Li, Siqi Wang, Jun Cao

**Affiliations:** ^1^Department of Anesthesiology, The First Affiliated Hospital of Chongqing Medical University, Chongqing 400016, China; ^2^Orthopedics Department, The First Affiliated Hospital of Chongqing Medical University, Chongqing 400016, China; ^3^Department of Pathology, School of Basic Medicine, Chongqing Medical University, Chongqing 400016, China

## Abstract

**Objective:**

To explore the related risk factors of postoperative delirium (POD) after hip or knee arthroplasty in elderly orthopedic patients and the predictive value of related risk factors. *Material and Methods*. In total, 309 patients (≥60 years) who received knee and hip arthroplasty between January 2017 and May 2020 were consecutively selected into the POD and nonpostoperative delirium (NPOD) groups. Group bias was eliminated through propensity score matching. Univariate and multivariable logistic analysis was used to determine the risk factors for POD. The nomogram was made by R.

**Results:**

58 patients were included in each group after propensity score matching; multivariable analysis demonstrated that LDH (OR = 4.364, *P* = 0.017), CHE (OR = 4.640, *P* = 0.004), Cystatin C (OR = 5.283, *P* = 0.006), arrhythmia (OR = 5.253, *P* = 0.002), and operation duration (OR = 1.017, *P* = 0.050) were independent risk factors of POD. LDH, CHE, Cystatin C, and arrhythmia were used to construct a nomogram to predict the POD. The nomogram was well calibrated and had moderate discriminative ability (AUC = 0.821, 95% CI: 0.760~0.883). Decision curve analysis demonstrated that the nomogram was clinically useful.

**Conclusions:**

Our study revealed that arrhythmia, operation duration, the increase of lactate dehydrogenase and Cystatin C, and the decrease of cholinesterase were reliable factors for predicting postoperative delirium after elderly hip and knee arthroplasty. Meanwhile, the nomogram we developed can assist the clinician to filtrate potential patients with postoperative delirium.

## 1. Introduction

Currently, knee and hip arthroplasty are taking up an increasing proportion of orthopedic surgery, and the demand especially from those patients mainly over 60 years old will continue to grow [1, 2]. Evidence has indicated that postoperative delirium (POD) is a relatively common and serious complication in patients undergoing hip and knee arthroplasty, and the probability of occurrence is up to 17.6% [3]. POD is an acute clinical reversible syndrome characterized by a typical dysfunction of the patient's cognition and attention after anesthesia and surgery [4]. It is worth noting that POD has a remarkable influence on prognosis and can even lead to worse outcomes, such as aggravative infection, delayed recovery time, and aggrandized postoperative mortality [5, 6].

Hence, it is extremely important to identify patients with potential risk of POD before surgery, which can help clinical decision-makers to achieve preventive effect through a variety of interventions during the perioperative period. At present, many risk factors have been identified, but the risk factors obtained from most studies are limited to demographic characteristics, such as patient's age, sex, and past history [7–10], while few studies on risk factors related to laboratory data, and rarely focus on knee and hip arthroplasty surgeries. In addition, few studies have constructed preoperative predictive models based on risk factors to predict the risk of POD.

In order to address the above limitations on POD, the purpose of this retrospective study was to identify risk factors with hip and knee arthroplasty surgery and to build preoperative predicting models to assist the clinician in determining the probability of POD and taking interventions to minimize the possibility of POD.

## 2. Material and Methods

Prior to data collection, the study was approved by the Ethics Committee of the First Affiliated Hospital of Chongqing Medical University (2021-201), and because all data were collected from the electronic medical record system, the requirement for informed consent was waived throughout the Ethics Committee's agreement. This manuscript adheres to the applicable STROBE guidelines.

We retrospectively reviewed 309 patients aged over 60 years who were from Orthopedics of the First Affiliated Hospital of Chongqing Medical University from January 2017 to May 2020.

*Inclusion criteria*: (I) aged over 60 years old; (II) elective surgery includes hip arthroplasty (unilateral or bilateral); (III) elective surgery includes knee arthroplasty (unilateral or bilateral, total or unicompartment).

*Exclusion criteria*: (I) incomplete medical records and lack of one or more laboratory indicators; (II) diagnosed in delirium before surgery; (III) noninitial joint arthroplasty surgery.

### 2.1. Anesthesia and Postoperative Analgesia

*Induction of anesthesia*: 1.5 mg/kg propofol + 0.5 *μ*g/kg sufentanil + 0.1 mg/kg vecuronium bromide. *Maintenance of anesthesia*: 1.5% sevoflurane + 9-12 *μ*g/kg/h propofol + 10-15 mg/kg/h remifentanil and intermittent administration of sufentanil for pain relief. *Analgesia*: patients routinely use PCNA (patient controlled nerve analgesia) for self-controlled analgesia after surgery, and the pain is controlled at mild pain (VAS score: at rest <3, at movement <4).

### 2.2. Delirium

Two orthopedic nurses trained in the assessment of delirium participated in the clinical evaluation of all joint replacement patients. They used the Confusion Assessment Method (CAM) which is suggested to diagnose POD to distinguish whether patients had postoperative delirium at the previous day and the first, second, and third postoperation days of joint replacement [11]. Based on the diagnosis after joint replacement, we divided them into the POD group and the nonpostoperative delirium (NPOD) group.

### 2.3. Data Collection

Clinical data and laboratory data were saved in Electronic Medical Record (Wining Net 5.0.)

The preoperative data include sex, age, past history (including smoking, drinking, diabetes, hypertension, and coronary heart disease), history of mental illness or psychotropic drug use, history of blood transfusion, glomerular filtration rate (GFR), C-reactive protein (CRP), lactate dehydrogenase (LDH), cholinesterase (CHE), Cystatin C, erythrocyte sedimentation rate (ESR), hemoglobin (HB), arrhythmia (including the abnormality of the frequency, rhythm, origin, conduction velocity, and activation sequence of cardiac impulses), ejection fraction (EF), left ventricular diastolic dysfunction (LVD, diagnosed by ASE/EACVI Guidelines and Standards [12]), white blood cell count (WBC), absolute neutrophil count (NE), lymphocyte count (LY), monocyte count (MO), eosinophil count (EO), basophil count (BA), total protein (TP), albumin (AL), total bilirubin (TBil), direct bilirubin (DBil), alanine transaminase (ALT), aspartate aminotransferase (AST), alkaline phosphatase (ALP), creatinine (Cr), blood urea nitrogen (BUN), calcium (Ca), and magnesium (Mg).

The intraoperative data include anesthesia, intraoperative blood loss, operation duration, surgical approach, and surgical grade.

### 2.4. Statistical Analysis

Propensity score matching (PSM) was applied to minimize the influence of confounding factors such as selection bias. Based on the propensity scores, postoperative delirium patients were matched in 1 : 1 ratio to normal patients using greedy nearest neighbor matching algorithm without replacement and match tolerance equal to 0.01. Refer to the previous study; when fitting the PSM model, 14 baseline characteristics which were proven to be risk factors of POD were used as baseline covariates to participate in the analysis: age, sex, smoking, drinking, diabetes, hypertension, coronary heart disease, history of mental illness or psychotropic drug use, blood transfusion, anesthesia, surgical approach, surgical grade, EF, and LVD [8, 13–15]. Standardized differences for categorical variables before and after PSM were evaluated by chi-square, but for the continuous variable, independent *T* test was used. We considered *P* > 0.05 as no statistical significance, which means the clinical feature did not differ between the two groups.

Univariate and multivariable analyses based on logistic regression were used to analyze independent risk factors for POD. Variables with a value of *P* ≤ 0.2 in univariate analysis would be put into multivariable analysis, and then, if *P* ≤ 0.05, the variables were considered as the independent risk factors of POD.

All patients were as a dataset to develop the nomogram, and preoperative variables that were statistically significant in the multivariable analysis were used to construct the nomogram. The receiver operating characteristic (ROC) curve with area under the curve (AUC) was used for discrimination capacity. The performance of the nomogram was assessed by a calibration plot for internal calibration. The decision curve analysis (DCA) was adopted to evaluate the clinical efficacy of the nomogram and analyze the net benefit under different risk thresholds in POD patients.

R was used to construct the nomogram model of risk assessment using the “foreign,” “rmda,” and “rms” packages. IBM SPSS version 25.0 was used for PSM analysis.

## 3. Results

Patients who underwent hip and knee arthroplasty in our hospital from 2017.01 to 2020.05 were included. 68 patients with postoperative delirium and 241 patients without postoperative delirium were selected into the POD group and the NPOD group, respectively. After data collection, 65 and 195 patients were eligible for the study and separately divided into the POD group and the NPOD group, respectively. 58 patients were included in each group after PSM. The research flow chart is shown in Figure 1.

### 3.1. Clinical Characteristics

Before PSM, there were 65 and 195 patients in the POD group and the NPOD group; the clinicopathological characteristics of the two groups of patients are summarized in Table 1. Elderly patients were more likely to have POD (*P* = 0.046). Those who received blood transfusion (*P* = 0.037) or hip replacement surgery (*P* = 0.031) were more likely to have POD. After PSM, there were no differences in the two groups in which each group had the same number of patients (all *P* > 0.05); the clinicopathological characteristics of the matched patients are revealed in Table 1.

### 3.2. Univariate and Multivariable Regression Analyses

Univariate analyses showed that operation duration (*P* < 0.2), LDH (*P* < 0.2), CHE (*P* < 0.2), Cystatin C (*P* < 0.2), arrhythmia (*P* < 0.2), NE (*P* < 0.2), TBil (*P* < 0.2), DBil (*P* < 0.2), Cr (*P* < 0.2), and Mg (*P* < 0.2) were significant. Multivariable analyses revealed that patients with higher LDH (OR = 4.364, *P* = 0.017), higher Cystatin C (OR = 5.283, *P* = 0.006), arrhythmia (OR = 5.253, *P* = 0.002), or lower CHE were more likely to have POD, and if patients experienced prolonged operation duration (OR = 1.017, *P* = 0.05), they were more likely to suffer POD than other patients (Table 2).

### 3.3. Nomogram Analysis

The nomogram was internally validated by computing the bootstrap-corrected Harrell index and by the calibration plot. The AUC of the model was 0.821 with a 95% CI ranging from 0.760 to 0.883, which shows that the model has strong predictive ability. And as illustrated in Figure 2, the nomogram was well calibrated and clinically useful.

For each patient, the total point was calculated by adding up the score of each variable to predict the opportunity of POD after orthopedic surgery. For each independent variable, we draw a straight line perpendicular to the axis of the variable, and the intersection with the “Points” represents the score of the independent variable. For example, CHE ≤ 5400 means a score of 100 and LDH < 250 means a score of 0. The total score of the corresponding points of these independent variables of the patient can be calculated, which will be positioned on the “Risk of POD” in a vertical line.

DCA clearly stated that if the threshold probability is between 12% and 95%, using the nomogram we developed to forecast POD of arthroplasty patients adds benefit than either the treat-all patients scheme or the treat-none scheme (Figure 3). For example, if the high-risk threshold probability of a patient is 30%, then the net benefit is 0.252 when using the nomogram to make the decision of whether to undergo treatment.

## 4. Discussion

POD has long been acknowledged as a significant complication in surgery patients. With the aging of the population and the increase of joint diseases, the demand for joint replacement surgery is also increasing [16]. Studies have shown that the incidence of POD after major surgery is 20% to 50% in people over the age of 60 [17].

Previous abundant studies have identified multiple risk factors notably related with POD, including age, sex, drinking, smoking, cognitive impairment, higher blood glucose, hypertension, renal function, and cardiac function [3, 15, 18, 19]. Hence, we used the patient's past history and the related clinical indicators as the matching baseline for PSM analysis.

In this retrospective study, we found that preoperative arrhythmia, operation duration, increase of LDH and Cystatin C, and decrease of CHE were independent risk factors for POD; simultaneously, the nomogram was a reliable tool for clinical decision-makers to predict the development of POD.

Operation duration has been identified as a risk factor for POD in numerous studies [20–22]. We came to the same conclusion throughout multiple analyses. There is no doubt that long operation duration results in prolonging anesthesia time and surgical stimulation time which may cause acute stress and aggravate the inflammatory reaction. Therefore, operation duration increases the risk of POD for patients. Meanwhile, the “operation duration” in our study is simple duration from the beginning of the operation to the end of the operation. In fact, we deem that the whole time of severe surgical injury stimulus may be the pivotal reason of POD, because severe surgical injury stimulus leads to greater acute inflammatory reaction than general surgical procedure (such as separate organization), which explains the higher incidence of delirium after hip, knee, and heart surgery.

In a cohort study, Cerejeira et al. found that patients with postoperative delirium had decreased levels of acetylcholinesterase before operation [23]. From a systems neuroscience perspective, some scholars have believed that the pathogenesis of postoperative delirium is due to the neurotransmitter imbalances particularly involving dopamine and acetylcholine [17, 24]. Nevertheless, as a clinical laboratory index that can reflect liver function, LDH has not been reported as an independent risk factor for POD. It is a routine examination before operation, and abnormal increase is considered to be a vigilant factor for liver function damage [25]. We suspect that the damage of liver function leads to the slow metabolism of anesthetic drugs, which made the drugs accumulate in the body, affecting the brain function and causing cognitive impairment after operation. The mental abnormality caused by this metabolic disorder will continue to inhibit or excite the brain function until it returns to normal after the complete metabolism of the drug.

Also, to our knowledge, Cystatin C has not been mentioned as an independent risk factor for POD in previous articles. However, it is mentioned in some articles that the decline of renal function is the cause of POD. As a routine indicator of renal function, the measurement of GFR is often affected by muscle mass. Due to physical weakness, GFR in elderly patients has difficulty in reflecting the real renal function before operation and even overestimates renal metabolic function, while Cystatin C is not affected by age, sex, weight, and inflammatory reaction, so Cystatin C can more sensitively capture the changes of renal function [26]. The kidney is the main pathway of perioperative metabolism of some drugs, especially anesthesia-related drugs. With the increase of age, renal function begins to decline, which reduces the metabolic capacity of drugs, which may also cause the accumulation effect of drugs [27]. Moreover, the ability of renal hypofunction patients to rely on renal blood pressure regulation becomes worse, resulting in intraoperative retention of sodium and water, excessive circulation volume leads to tissue cell edema, and the ability to obtain oxygen is weakened. This may be a cause of postoperative brain dysfunction [28].

Other studies have shown that the increase of preoperative CRP and the decrease of preoperative total protein, albumin, and hemoglobin are independent risk factors for postoperative delirium, which contradicts our conclusions [13, 14, 18, 20]. We speculate that this is due to the fact that we use the PSM method to control the confounding factors and eliminate the interference [29]. In the study of Ren et al., they found that the increase of CRP is the independent risk of POD [30]; the difference is that they use the change of CRP (values of serum CRP between before and after surgery) as a variable, rather than a simple preoperative CRP value. We believe that the cause of POD should be the increasing inflammatory reaction during operation, not the inflammatory state before operation, and some studies have also found proinflammatory factors in the cerebrospinal fluid of patients with postoperative delirium [31], so the increase of preoperative CRP (or ESR) does not prove that patients have the risk of POD, but attention should be paid to the dynamic fluctuation of inflammatory indexes in perioperative patients.

In recent years, many models for predicting POD have been mentioned in a few studies [32, 33]. Compared to individual risk factors, the predictive model based on several risk factors is further capable in assisting the clinician in noticing the patients who are prone to POD. Zhang et al. built a model on the basis of preoperative cognitive impairment, multiple medical comorbidities, ASA classification, transfusion > 2 units of red blood cell, and intensive care, but their model showed an inferior C-index of 0.67 (95% CI 0.62-0.72) [33]. In addition, the evaluation of risk factors brought into the model was subjective, which would deeply reduce the final prediction effect of the model. Therefore, we presented and validated a nomogram, which is constructed by preoperative variables. Clinical workers, even patients, can utilize this model to estimate the risk of suffering POD and make preparations accordingly.

This retrospective study still had some limitations. First, due to the limitations of the conditions, this study mainly collects the preoperative laboratory test results, so the intraoperative and postoperative test results cannot be included in the study. Second, we only assess delirium for patients three days after operation, but present POD assessment should be extended to the seventh day after operation, so there is a certain probability of missed diagnosis for the patients with postoperative delirium. Third, although PSM was used to balance the bias between two groups, there may still be potential factors that affected the results, and our study is mainly aimed at elderly orthopedic patients undergoing hip or knee arthroplasty, and whether the conclusion can be applied to other populations needs to be further verified.

## 5. Conclusion

Our study found that preoperative arrhythmia, operation duration, increase of LDH and Cystatin C, and decrease of CHE were independent risk factors for delirium after elderly orthopedic hip and knee arthroplasty. The nomogram constructed by LDH, CHE, Cystatin C, and arrhythmia can assess the risk of postoperative delirium in patients undergoing hip and knee arthroplasty.

## Figures and Tables

**Figure 1:** Flow diagram of the study patients. POD: postoperative delirium.

**Figure 2:** (a) Nomogram model predicts the probability of POD. (b) Calibration plot of the nomogram. The nomogram was calibrated for the probability of being POD (bootstrap 1000 repetitions). (c) The discrimination assessed by ROC curve. The AUC is 0.821 (95% CI 0.760~0.883). POD: postoperative delirium; ROC: receiver operating characteristic; AUC: area under the curve; CI: confidence interval.

**Figure 3:** Decision curve analysis (DCA) for nomogram established to predict POD. The *y*-axis measured the net benefit. The thick black line represents the net benefit of no patient suffering POD. The thin grey line shows the net benefit of all patients suffering POD.

**Table 1:** Baseline characteristics of before and after PSM.

Characteristics	Before PSM			After PSM		
	POD (65)	NPOD (195)	*P* value	POD (58)	NPOD (58)	*P* value
Mean (SD) age (years)	85.06 ± 7.04	82.77 ± 8.29	**0.046**	84.93 ± 6.40	86.16 ± 6.50	0.309
Sex (%)			0.806			0.656
Male	16 (24.6)	51 (26.2)		14 (24.1)	12 (20.7)	
Female	49 (75.4)	144 (73.8)		44 (75.9)	46 (79.3)	
Smoking (%)			0.439			1
Yes	6 (9.2)	25 (12.8)		6 (10.3)	6 (10.3)	
No	59 (91)	170 (87.2)		52 (89.7)	52 (89.7)	
Drinking (%)			0.166			0.508
Yes	4 (6.2)	24 (12.3)		4 (6.9)	6 (10.3)	
No	61 (93.8)	171 (87.7)		54 (93.1)	52 (89.7)	
Diabetes (%)			0.328			0.573
Yes	20 (30.8)	48 (24.6)		18 (31.0)	15 (25.9)	
No	45 (69.2)	147 (75.4)		40 (69.0)	43 (74.1)	
Hypertension (%)			0.430			0.71
Yes	32 (49.2)	107 (54.9)		30 (51.7)	28 (48.3)	
No	33 (50.8)	88 (45.1)		28 (48.3)	30 (51.7)	
Coronary heart disease (%)			0.928			0.498
Yes	13 (20.0)	38 (19.5)		11 (19.0)	14 (24.1)	
No	52 (80.0)	157 (80.5)		47 (81.0)	44 (75.9)	
Mental illness or psychotropic drug use (%)			0.068			1
Yes	10 (15.4)	15 (7.7)		5 (8.6)	5 (8.6)	
No	55 (84.6)	180 (92.3)		53 (91.4)	53 (91.4)	
Blood transfusion (%)			**0.037**			1
Yes	20 (30.8)	36 (18.5)		14 (24.1)	14 (24.1)	
No	45 (69.2)	159 (81.5)		44 (75.9)	44 (75.9)	
Anesthesia (%)			1			1
General anesthesia	65 (100.0)	195 (100.0)		58 (100.0)	58 (100.0)	
Others	0 (0)	0 (0)		0 (0)	0 (0)	
Surgical approach (%)			**0.031**			0.170
Hip replacement	61 (93.8)	162 (83.1)		54 (93.1)	57 (98.3)	
Knee replacement	4 (6.2)	33 (16.9)		4 (6.9)	1 (1.7)	
Surgical grade (%)			0.102			0.782
3	57 (87.7)	153 (78.5)		50 (86.2)	51 (87.9)	
4	8 (12.3)	42 (21.5)		8 (13.8)	7 (12.1)	
Mean (SD) ejection fraction	64.80 ± 3.65	61.65 ± 3.80	0.776	64.91 ± 3.72	65.29 ± 4.02	0.599
Left ventricular diastolic dysfunction (%)			0.474			0.298
Yes	57 (87.7)	177 (90.8)		52 (89.7)	55 (94.8)	
No	8 (12.3)	18 (9.2)		6 (9.3)	3 (5.2)	

Significant *P* values are in bold (*P* < 0.05). SD: standard deviation; PSM: propensity score matching; POD: postoperative delirium.

**Table 2:** Risk factors of patients with POD by univariate and multivariable based on logistic regression analysis.

Characteristic	Univariate analyses		Multivariate analyses	
	OR (95% CI)	*P* value	OR (95% CI)	*P* value
Intraoperative blood loss	1.002 (0.997-1.007)	0.404	—	—
Operation duration	1.013 (0.999-1.026)	0.063^a^	1.017 (1.000-1.035)	**0.050**
Glomerular filtration rate	1.274 (0.484-3.353)	0.623	—	—
C-reactive protein	0.655 (0.264-1.625)	0.361	—	—
Lactate dehydrogenase	2.450 (0.994-6.042)	0.052^a^	4.364 (1.295-14.707)	**0.017**
Cholinesterase	4.107 (1.813-9.305)	0.001^a^	4.640 (1.654-13.013)	**0.004**
Cystatin C	4.950 (2.525-10.882)	<0.001^a^	5.283 (1.603-17.415)	**0.006**
Erythrocyte sedimentation rate	1.000 (0.472-2.117)	1.000	—	—
Hemoglobin	1.158 (0.547-2.453)	0.702	—	—
Arrhythmia	3.528 (1.612-7.720)	0.002^a^	5.253 (1.870-14.756)	**0.002**
White blood cell count	1.435 (0.622-3.315)	0.397	—	—
Absolute neutrophil count	1.630 (0.781-3.404)	0.193^a^	2.152 (0.804-5.761)	0.127
Lymphocyte count	0.000	0.999	—	—
Monocyte count	0.812 (0.391-1.687)	0.576	—	—
Eosinophil count	0.491 (0.043-5.572)	0.566	—	—
Basophil count	1.000	1.000	—	—
Total protein	1.231 (0.593-2.554)	0.577	—	—
Albumin	0.924 (0.423-2.017)	0.842	—	—
Total bilirubin	3.062 (1.014-9.248)	0.047^a^	1.240 (0.199-7.711)	0.817
Direct bilirubin	1.829 (0.749-4.462)	0.185^a^	1.150 (0.251-5.269)	0.858
Alanine transaminase	0.482 (0.085-2.742)	0.411	—	—
Aspartate aminotransferase	0.590 (0.181-1.923)	0.381	—	—
Alkaline phosphatase	0.000	0.999	—	—
Creatinine	2.115 (0.938-4.773)	0.071^a^	0.705 (0.206-2.414)	0.578
Blood urea nitrogen	1.725 (0.741-4.014)	0.206	—	—
Calcium	1.573 (0.614-4.032)	0.346	—	—
Magnesium		0.120^a^		0.559
Lower	1		1	
Normal	1 (0.073-13.644)		3.070 (0.139-67.724)	
Raised	0.284 (0.029-2.824)		1.347 (0.088-20.677)	

^a^Represents the significant *P* value of univariate analysis (*P* < 0.2); significant *P* values of multivariate analyses are in bold (*P* ≤ 0.05). POD: postoperative delirium.

## Data Availability

The data of this manuscript are available from the corresponding author on reasonable request.
